# An Improved Logistic Regression Method for Assessing the Performance of Track and Field Sports

**DOI:** 10.1155/2022/6341495

**Published:** 2022-08-02

**Authors:** Songling Zheng, Xi Man

**Affiliations:** Institute of Physical Education, Inner Mongolia Normal University, Hohhot 010020, China

## Abstract

Track and field is an important part of sports. Track and field athletes are an important reserve force for the development of national sports. An accurate assessment of track and field athletes' performance can help them develop more appropriate training programs and improve their performance. In order to assess the performance of track and field athletes better, this paper proposes an improved logistic regression method. Firstly, this method uses factor analysis to reduce the data dimensions of the factors that affect the performance of track and field athletes, and uses the principal component analysis to select common factors and their corresponding values. Then, according to the common factors, a binary logistic regression model is established to evaluate the performance of track and field athletes. Experiments show that the method can effectively evaluate the performance of track and field athletes and is suitable for athletes of different track and field sports. It has high accuracy, fast evaluation efficiency, and good universality of performance evaluation. For different numbers of athletes, the proposed method has a lower error evaluation index, higher evaluation accuracy, and better evaluation quality. Compared with the other two methods, the proposed method has the shortest evaluation time and is more effective for the performance evaluation of track and field athletes.

## 1. Introduction

Athletes are an important reserve force for the development of national sports, and the accurate assessment of athletes' performance can develop more applicable training plans for them and improve their performance [1]. In addition to a complete training system, an objective and fair assessment evaluation system is particularly important for training athletic sports talents. An objective evaluation system of track and field sports performance aims to explore the potential of track and field athletes and is conducive to the national selection of more suitable track and field sports talents [2]. Constructing an evaluation model reflects the objective training effects of track and field athletes, finds the strengths and weaknesses of track and field athletes themselves, and then promotes track and field training reform and maximizes the effects and benefits of the sports training reform. At the same time, the feedback information from the model can also promote track and field athletes to clearly recognize their training situation in the future training process and continuously adjust their training status to achieve the highest training efficiency. This can also serve as a guideline for track and field athletes' career planning.

Factors such as training intensity and track and field athletes' own physical quality can directly affect their performance. Accurately understanding the changing characteristics of track and field athletes' performance can ensure their better performance [3]. This makes it very important to assess track and field athletes' performance. The assessment of track and field athletes' performance is an important part of the athletes' training activities. This work plays a role in diagnosing, regulating, and strengthening the training process of track and field athletes, as well as making value judgments about the effectiveness of their training [4]. The evaluation of the training effectiveness of track and field athletes should be an evaluation of the training effect and training process. The evaluation should not only emphasize the function of screening and selection, but also strengthen the function of motivation and development [5]. What should we do in the evaluating the training performance of track and field athletes to achieve the purpose of cultivating the training interest of track and field athletes, stimulating the subjective initiative of track and field athletes, and meeting the psychological needs of athletes is directly related to the functional orientation of track and field athletes' training and the realization of training goals. This is a problem that needs to be solved urgently at present.

Athletic athlete performance assessment is not only a test of sports training effects, but also a comprehensive judgment of athletes' sports ability. Whether the assessment is comprehensive, objective and fair, and truly reflects an athlete's actual level in sports [6] is often an concern of the athletes. Therefore, it is particularly important to construct a diversified performance assessment system. The diversification of the assessment system is reflected in the diversification of the assessment content. Athletic performance assessment should not be limited to physical fitness and motor skills, but also include training attitude, physical exercise, training participation, and competition winning together. The assessment should cover various factors such as cognition, emotion, cooperation, learning, and practice of the athletes [7]. The diversification of the assessment system is also reflected in the setting of dual subjects of assessment. They are the summative assessment made by the coach as the main body relying on the assessment results of training programs and the formative assessment made by the athlete as the main body with training activities as the main content [8]. By constructing a diversified track and field athletes' performance assessment system, it further broadens the dimensions and connotations of track and field athletes' performance assessment, which is of practical significance to improve the fairness and comprehensiveness of track and field athletes' performance assessment, enhance track and field athletes' participation and dominance in the process of performance formation, and help track and field athletes understand themselves, discover themselves, and transform themselves more objectively.

The regression model is a predictive model that studies the dependent and independent variables and integrates various possible influencing factors to assess athletes' performance and training effects through multiple regression models [9]. The research methodology in this paper takes the factors affecting the training performance of track and field athletes as the object of study, selects the factors affecting the assessment of track and field athletes' performance as the target variable, and establishes a logistic regression model. In this paper, the historical performance of track and field athletes was selected as the dataset. Among the assessment variables were competition ranking, competition time, age, gender, training duration, BMI, and blood pressure. First, factor analysis is carried out on the evaluation indicators to reduce the dimension of the data, eliminate the correlation between the data, and determine the final indicators. Then, a logistic regression model was established based on the final indicators. Finally, the assessment effects of the models were compared. Compared with the other methods, the method in this paper can achieve high-quality assessment of track and field athletes' performance, which is very important for their training planning. Accurate assessment of track and field athletes' performance can help them understand themselves and training planning, which is good to improve their performance and make them better and better.

This paper has the following innovative points.

1. The factors affecting track and field athletes' performance are multiple. In order to effectively conduct track and field athletes' performance assessment, this paper simplifies the data and influencing factors by the factor analysis method. Discarding secondary factors and selecting primary factors as evaluation variables allows for a more simplified and efficient operation of the algorithm.
2. The common factors affecting the performance of track and field athletes were selected using the principal component analysis, and classified and assigned different weight values according to the degree of influence, which can improve the accuracy of the evaluation.

This paper mainly consists of five parts; the first is the introduction, the second is the state of the art, the third is the methodology, the fourth is the experiment and analysis, and the fifth is the conclusion.

## 2. State of the Art

### 2.1. Research Status

At present, with the deepening of the concept of “Internet Plus,” information technology has been widely used in sports training activities. A large number of scholars have conducted in-depth research on sports performance assessment models and constructed many assessment models. Under the guiding principles of advancement and comprehensiveness, the literature [10] established indicators such as training hours to improve the quality of sports training and to promote further the internalization of athletes' knowledge. The literature [11] established an evaluation model from three aspects of the basic needs theory. The model used hierarchical analysis to analyse the indicator weights and found that the greatest weight was given to the autonomy needs and the least weight to the competence needs. When summarizing the methodological studies on the quantification of performance evaluation in universities, hierarchical analysis was found to be the most representative, but it is very difficult to test whether the judgment matrix is consistent when studying real-world problems and it is difficult to truly reflect the fuzzy nature of human evaluation [12]. Therefore, the literature [13] addresses the shortcomings of expert scoring in the hierarchical analysis method and integrates the principles of fuzzy mathematics to establish a mathematical model to evaluate the training quality more objectively. The literature [14] established an evaluation system from three aspects: training platform, coaches, and athletes. The method is based on AHP to determine the index weights and introduces a fuzzy comprehensive evaluation model for the differences that exist between the consistency of judgment matrix and the consistency of human brain thinking. This provides a new perspective for athlete training quality assessment. With the continuous improvement of the fuzzy complementary judgment matrix theory, the literature [15] established athlete satisfaction indicators. The theory indicates that the influence of personal factors on the index system is the highest and the influence of gymnasium factors is the lowest, which provides a more scientific and reasonable reference basis for athlete training strategies. The literature [16] investigated the athlete performance prediction method integrating knowledge mapping and collaborative filtering to establish a training knowledge map depicting training information. The algorithm calculates the similarity of training at the knowledge level by the neighbour node-based method and the knowledge graph-based learning method, and integrates the obtained similarity into the collaborative filtering performance prediction framework to obtain athlete performance prediction results. The literature [17] investigates a two-way attention-based mechanism for athlete performance prediction model. The model obtains the attention scores of different attribute features on the first stage and second stage competition performance through two attention calculations, and combines the multi-feature fusion approach to obtain the competition performance prediction results. The historical data-driven prediction method is implemented by historical data. There are many historical data-driven prediction methods such as hidden Markov models, chaotic prediction, and support vector machines [18]. Support vector machines have the advantage of small sample learning and high learning ability in prediction, and hence they are also used to study the historical data-driven athlete performance estimation method. This method uses the KNN algorithm to pre-process the historical performance of athletes to remove the effect of distracting data and classify the data accurately. It uses support vector institutions to build regression prediction models and introduces Lagrangian functions for data transformation to avoid data operations from getting localized [19]. The support vector regression prediction model parameters are optimized using the particle swarm algorithm to reduce the interference of input quantity noise and reduce the complexity of the computation. These evaluation models are built according to different application scenarios and are important for promoting the scientific training of athletes.

### 2.2. Factor Analysis Method

Factor analysis is a technique to reduce the dimensionality and simplify the data. It explores the underlying structure of the observed data by examining the internal dependencies among many variables and represents the underlying data structure with a few “abstract” variables. These abstract variables are called “factors.” By discarding secondary factors and selecting primary factors as evaluation variables, the model is made more simplified and the efficiency of the algorithm operation is improved. This reflects the main information of the original set of variables. The original variables are observable explicit variables, while the factors are generally unobservable latent variables. The common factors in factor analysis are common influences that are not directly observable but exist objectively. Each variable can be expressed as a linear function of the common factor and the sum of the special factors [20]. Its mathematical model can be expressed as

(1) $$\begin{array}{c} \left(\begin{array}{c} i_{1}\\ i_{2}\\ \vdots \\ i_{u} \end{array}\right)=\left(\begin{array}{ccc} g_{11} & L & g_{1u}\\ g_{21} & \cdots & g_{2u}\\ \vdots & \; & \vdots \\ g_{u1} & \cdots & g_{uw} \end{array}\right)\left(\begin{array}{c} F_{1}\\ F_{2}\\ \vdots \\ F_{w} \end{array}\right)+\left(\begin{array}{c} \varepsilon_{1}\\ \varepsilon_{2}\\ \vdots \\ \varepsilon_{w} \end{array}\right). \end{array}$$

That is, *I* *=* *GF* *+* *ε*, where *I*=(*i*_1_, *i*_2_,…,*i*_*u*_)^*N*^ is an observable *u-dimensional* random vector. Each component represents an indicator or vector. *F* in *F*=(*F*_1_, *F*_2_,…,*F*_*w*_)^*N*^ is an *w-common factor* variable. *w* is less than or equal to *u*. It is the factor that appears in the expressions of each original observed variable, which are mutually independent unobservable theoretical variables. Matrix *G* is called the factor loading matrix. *g*_*xy*_ is called the factor loading. It represents the correlation coefficient between the *x-th* original variable and the *y-th* public factor variable. The larger *g*_*xy*_ indicates the stronger correlation between the public factor *F*_*y*_ and the original variable *I*. *ε* is a special factor. It represents the part of the original variables that cannot be explained by the common factor variables, which is equivalent to the residual part in the multiple linear regression analysis.

Factor analysis utilizes the idea of dimensionality reduction, starting from the study of the dependencies within the correlation matrix of the original variables, and groups the original variables according to the magnitude of the correlation, making the correlation between variables within the same group high and the correlation between variables in different groups low [21]. Each group of variables represents a basic structure and is represented by an unobservable composite variable. This underlying structure is called the common factor. Capturing these main factors can help us analyse and interpret complex problems.

## 3. Methodology

### 3.1. Regression Models

#### 3.1.1. Regression Model Where the Dependent Variable Is a Qualitative Variable

*(1) Qualitative variables* The dependent variable takes only two outcomes. *j* *=* *0* means that the event did not occur. *j* *=* *1* means that the event occurred. Consider the following expression for a simple linear regression model.

(2) $$\begin{array}{c} j_{x}=\beta_{0}+\beta_{1}i_{x}+\varepsilon_{x},\\ E\left(j_{x}\right)=\beta_{0}+\beta_{1}i_{x}. \end{array}$$

Since *j*_*x*_ is a Bernoulli random variable of type 0 to 1, the following probability expression is obtained:

(3) $$\begin{array}{c} U\left(j_{x}=1\right)=\pi_{x},\\ U\left(j_{x}=0\right)=1-\pi_{x}. \end{array}$$

According to the definition of discrete random variable expectation, the following function is obtained:

(4) $$\begin{array}{c} E\left(j_{x}\right)=1\left(\pi_{x}\right)+0\left(1-\pi_{x}\right)=\pi_{x}. \end{array}$$

Thus,  *E*(*j*_*x*_)=*π*_*x*_=*β*_0_+*β*_1_*i*_*x*_.

*(2) Error term* The error term *ε*_*x*_=*j*_*x*_ − (*β*_0_+*β*_1_*i*_*x*_) can only take two values for a dependent variable, i.e., 0 or 1. Its expression is as follows:

(5) $$\begin{array}{c} j_{x}=1,\varepsilon_{x}=1-\left(\beta_{0}+\beta_{1}i_{x}\right)=1-\pi_{x},\\ j_{x}=0,\varepsilon_{x}=-\left(\beta_{0}+\beta_{1}i_{x}\right)=-\pi_{x}. \end{array}$$

The error term is a two-point discrete distribution, and thus it cannot be assumed to be a normal error regression model.

Zero-mean heteroskedasticity means that the error term is zero-mean and its variances are not equal, and the expressions are as follows:

(6) $$\begin{array}{c} D\left(\varepsilon_{x}\right)=D\left(j_{x}\right)=\pi_{x}\left(1-\pi_{x}\right)=\left(\beta_{0}+\beta_{1}i_{x}\right)\left(1-\beta_{0}-\beta_{1}i_{x}\right). \end{array}$$

If a multiple linear regression equation is used to analyse the quantitative relationship between the dependent variable and the independent variable, the relationship function is expressed as follows:

(7) $$\begin{array}{c} j=\beta_{0}+\beta_{1}i_{1}+\beta_{2}i_{2}+\cdots +\beta_{w}i_{w}. \end{array}$$

(3) The left side of the equation *j* takes 0 or 1, and the right side of the equation can take any real number; the left and right sides do not correspond to each other in terms of the range of values. Therefore, multiple linear regression cannot be used for fitting the dependent variable as a qualitative variable.

#### 3.1.2. Logistic Regression Model

The logistic function has the form [22].

(8) $$\begin{array}{c} f\left(i\right)=\frac{e^{i}}{1+e^{i}}=\frac{1}{1+e^{-i}}. \end{array}$$

The range of values of its independent variable is (-∞,+∞) and the range of values of the function is (0,1).

The dependent variable *j* itself takes only two discrete values of 0 or 1. It is not suitable as the dependent variable in the regression model, such that

(9) $$\begin{array}{c} \pi_{x}=f\left(i_{x}\right)=\frac{1}{1+\exp\left(-\left(\beta_{0}+\beta_{1}i_{x}\right)\right)},\\ \ln\left(\frac{\pi_{x}}{1-\pi_{x}}\right)=\beta_{0}+\beta_{1}i_{x}, \end{array}$$

where *π*_*x*_ is the probability that the random variable *j* takes 1, and its value varies continuously in the interval [0, 1]; thus, *π*_*x*_ can be used as the dependent variable instead of *j*.

Let *j* be a variable of type 0 to 1, and *t* sets of observations be (*i*_*x*1_,…, *i*_*xu*_, *j*_*x*_), where *j*_*1*_,*j*_*2*_,…,*j*_*t*_ is a random variable that takes the value 0 or 1. The expression for the expected value is as follows:

(10) $$\begin{array}{c} E\left(j_{x}\right)=\pi_{x}=f\left(\beta_{0}+\beta_{1}i_{x1}+\cdots +\beta_{u}i_{xu}\right). \end{array}$$

The expression of the function for the logistic regression model [23] is as follows:

(11) $$\begin{array}{c} \pi_{x}=f\left(i_{x}\right)=\frac{e^{\beta_{0}+\beta_{1}i_{x1}+\cdots +\beta_{u}i_{xu}}}{1+e^{\beta_{0}+\beta_{1}i_{x1}+\cdots +\beta_{u}i_{xu}}}. \end{array}$$

Thus, *j*_*x*_ is a random variable of type 0 to 1 with mean *π*_*x*_=*f*(*β*_0_+*β*_1_*i*_*x*1_+⋯+*β*_*u*_*i*_*xu*_).; and the probability function is

(12) $$\begin{array}{c} U\left(j_{x}=1\right)=\pi_{x},\\ U\left(j_{x}=0\right)=1-\pi_{x}. \end{array}$$

The random probability of *j*_*x*_ can be defined as:

(13) $$\begin{array}{c} U\left(j_{x}\right)=\pi_{x}^{j_{x}}{\left(1-\pi_{x}\right)}^{1-j_{x}},j_{x}=0,1;x=1,\ldots ,t. \end{array}$$

The likelihood function of *j*_*1*_,*j*_*2*_,…,*j*_*t*_ is thus

(14) $$\begin{array}{c} L=\prod_{x=1}^{t}U\left(j_{x}\right)=\prod_{x=1}^{t}\pi_{x}^{j_{x}}{\left(1-\pi_{x}\right)}^{1-j_{x}}. \end{array}$$

The likelihood function is taken logarithmically and the following expression can be obtained:

(15) $$\begin{array}{c} \ln\;L=\sum_{x=1}^{t}\left[j_{x}\ln\;\pi_{x}+\left(1-j_{x}\right)\ln\left(1-\pi_{x}\right)\right]=\sum_{x=1}^{t}\left[j_{x}\ln\frac{\pi_{x}}{1-\pi_{x}}+\ln\left(1-\pi_{x}\right)\right]. \end{array}$$

Bringing equation (2.14) into the equation gives the expression

(16) $$\begin{array}{c} \ln\;L=\sum_{x=1}^{t}\left[\begin{array}{c} j_{x}\left(\beta_{0}+\beta_{1}i_{x1}+\cdots +\beta_{u}i_{xu}\right)-\\ \ln\left(1+\exp\left(\beta_{0}+\beta_{1}i_{x1}+\cdots +\beta_{u}i_{xu}\right)\right) \end{array}\right]. \end{array}$$

The maximum likelihood estimation yields the estimate $\;{\hat{\beta }}_{0},{\hat{\beta }}_{1},\ldots ,{\hat{\beta }}_{u}$ of *β*_0_, *β*_1_,…, *β*_*u*_.

### 3.2. Prediction Model

#### 3.2.1. Data Processing

The data taken in this paper are from the historical performance of athletes in a sports school. They mainly contain factors such as competition ranking, competition sports time, age, gender, training hours, and physical fitness at all levels of events. The dataset contains data related to 100 athletes. The dataset consists of training predictor variables and one target variable for track and field sports. The predictor variables include athletic athletes' competition ranking, competition time, age, gender, training time, BMI, and blood pressure, and the variable descriptions are shown in Table 1. The goal of the dataset is to predict athletic athletes' performance based on certain parameter measures contained in the dataset.

The process of data cleaning requires the consideration of the following effects.

1. Duplicate or irrelevant data.
2. Mislabelled data or multiple occurrences of the same label.
3. Missing or empty data points.
4. Outlier values.

The data are a standard database, and hence there is no duplicate or irrelevant data and no vacant data points have been checked. Since blood pressure, age, and body mass index cannot be 0 in general, and 0 is an abnormal data point, the rows with 0 values in each feature of blood pressure, age, and body mass index were filtered out. There were 724 valid data left after processing.

#### 3.2.2. Factor Analysis

*(1) Applicability Test of Factor Analysis*. The results of the KMO and Bartlett's sphericity tests on the data of track and field athletes using SPSS software are shown in Table 2. It is generally considered that if the KMO measure is greater than 0.5, then factor analysis can be performed. The significance of *p* = 0 indicates that there is a certain correlation between the original variables, and the conditions for factor analysis are available.

*(2) Extraction of Common Factors*. Factor analysis was performed on the data, and the extraction of principal components was performed by principal component analysis. Classifying them according to the degree of influence and assigning different weight values improves the assessment accuracy. Under the principle of eigenvalue of 1, three principal factors were retained, i.e., the seven variables were grouped into three categories. This reduces the amount of operations, but categorization causes information loss, and the amount of information retained is 64.49%, and the amount of information lost is large; thus, a common factor is added to make the amount of information lost reside within an acceptable range. The following variance interpretation Table 3 shows that each principal component contains the total variance of each original variable, and the improved retained information is 77.08%.

*(3) Public Factor Naming*. The original factor loading matrix was rotated by extracting the four public factors and performing maximum variance orthogonal rotation to obtain the variance maximum orthogonal rotation matrix, as shown in Table 4.

Based on the rotated component matrix, the four common factors can be named. The first factor Z1 has large loadings on the gender and age indicators. The second factor Z2 has larger loadings on the race ranking and race time indicators. The third factor Z3 has a large loading on BMI and training duration. The fourth factor Z4 has a larger loading on blood pressure. It can be found that the evaluation indexes corresponding to Z1 are indirect influence data. The evaluation indexes corresponding to Z2 are race performance-related data. The evaluation indexes corresponding to Z3 are other physical data. Z4 represents blood pressure. They are named as indirect factors, competition performance, physical quality, and blood pressure, respectively.

#### 3.2.3. Binary Logistic Regression

*(1) Hosmer-Lemeshaw test*. The original hypothesis H0: the model fits well with the observations. The results are shown in Table 5*p* = 0.279 > 0.05; the original hypothesis is accepted and the regression model can fit the data well.


(17) $$\begin{array}{c} \text{Logit}U=-0.82+0.65k_{1}+0.86k_{2}+0.67k_{3}+0.38k_{4}, \end{array}$$

(2) As shown in Table 7, the significant *p*-values are all 0, indicating that BMI, age, gender, and training duration have highly significant effects on the performance of track and field athletes. The effects were ranked from the highest to the lowest: BMI > age > gender > training duration.

(3) As shown in Table 7, the significant *p*-values are all 0, indicating that BMI, age, gender, and training duration have highly significant effects on the performance of track and field athletes. The effects were ranked from the highest to the lowest: BMI > age > gender > training duration.

(4) The accuracy is shown in Table 6, with an accuracy of 74.9%, which indicates that the model predicts more accurately.

(5) From the regression analysis of multiple factors, a binary logistic regression equation was established.where *U*=*β*_0_+*β*_1_*i*_1_+*β*_2_*i*_2_+⋯+*β*_*w*_*i*_*w*_.

## 4. Result Analysis and Discussion

Using track and field athletes of a sports school as the experimental subjects, 10 groups of 200m sprinters were randomly selected as the research subjects. The evaluation results are shown in Figure 1. According to Figure 1, the method of this paper can effectively evaluate the performance of 200m sprinters, and the estimated value is very close to the actual value. The experiment proves that the method in this paper can accurately estimate the performance of track and field athletes and has a high accuracy of track and field athletes' performance assessment results.

The athletes of 10 types of track and field sports were randomly selected in this sports school to verify the generality of this paper's method. Using the method of this paper, the athletes' performance of these 10 types of track and field sports was evaluated and compared with the actual values, and the evaluation accuracy of the 10 types of track and field sports is shown in Figure 2. According to Figure 2, it can be seen that for different types of track and field sports, the method in this paper can accurately assess the performance of track and field athletes, and the estimation accuracy is basically maintained at more than 96%. The experiment proves that the method in this paper has good generality and a high estimation accuracy for different types of track and field sports.

Comparing the method of this paper with the methods in the literature [16] and literature [17] clearly indicates that the assessment of athletes' performance of the above-mentioned 10 types of track and field sports was implemented at the same time. The evaluation accuracy and evaluation efficiency of the three methods were tested by comparing, among which literature [16] is a student performance prediction method integrating knowledge mapping and collaborative filtering, and literature [17] is a student performance prediction model based on a two-way attention mechanism. The performance of 100 athletes in each type of track and field sports was selected for testing and the average value was taken to enhance the credibility of the experiment. The accuracy and assessment efficiency of the three methods for assessing athletes' performance in the 10 types of track and field sports are shown in Figures 3 and 4. According to Figure 3, it can be seen that for athletes of different types of track and field sports, the assessment accuracy of athletes' performance of this paper's method is significantly higher than the remaining two methods, and the average assessment accuracy of this paper's method is 97.7%, the average assessment accuracy of literature [16] is 81.8%, and the average assessment accuracy of literature [17] is 86.5%. The experiment proves that when assessing the performance of athletes in different types of track and field sports, the method in this paper has the highest assessment accuracy, which significantly reduces the estimation error of athletes' performance and increases the credibility of the assessment results at the same time.

According to Figure 4, for athletes of different types of track and field sports, the evaluation time of this paper's method is significantly lower than the remaining two methods, and the evaluation time of this paper's method is always maintained within 20s with less variation, while the estimation time of the remaining two methods is more variable and less stable. This is due to the fact that the algorithm in this paper introduces factor analysis to optimize the parameters affecting the evaluation, which reduces the computational parameters and decreases the computational effort. The experiment proves that the evaluation time of this paper's method is the least and the athlete's performance evaluation is more efficient.

Taking 200m sprinters' performance as an example, the accuracy of the performance assessment of the three methods was tested with different numbers of athletes. The accuracy of the three methods was evaluated by the Mean Absolute Percentage Error (MAPE), an error evaluation index. The results of the error evaluation index tests for the three methods with different numbers of athletes are shown in Figure 5. According to Figure 5, the MAPE values of all three methods increased with the increasing number of athletes. Generally, if the MAPE value is lower than 10, it indicates that the evaluation accuracy of the evaluation methods is higher. With different numbers of athletes, the MAPE values of this paper are significantly lower than those of the remaining two methods. The MAPE value of this method always stayed within 6, and the MAPE value of the other two methods was lower than 10 only when the number of athletes was less than 200. When the number of athletes was more than 200, the MAPE values of the other two methods were greater than 10.

The experiment proves that the MAPE value of this paper method is the lowest when the number of athletes is different. This indicates that the evaluation value of this paper's method is closest to the actual value, with a higher evaluation accuracy and high evaluation quality.

## 5. Conclusion

Based on the model obtained in this paper, the performance of track and field athletes can be effectively evaluated. The main objective of this paper is to evaluate the performance of track and field athletes using a logistic regression model. The method adopts the idea of factor analysis, reduces and simplifies the data, and improves the evaluation effect. The experiments show that the method can accurately estimate the performance of track and field athletes and has a high accuracy of track and field athletes' performance assessment. At the same time, the method has good generality for track and field athletes' performance evaluation, less evaluation time, and higher evaluation efficiency. Overall, the method in this paper can achieve high-quality athlete performance assessment, which is very important for athletes' training planning. The accurate estimation of athletes' performance can help improve their performance and make them better by understanding the training planning they need. Therefore, we study the historical data-driven athlete performance estimation method to improve the accuracy and estimation efficiency of athlete performance estimation, provide more valuable information for athlete training planning, and develop better athletes for the country. However, the good experience of using this method requires a large amount of track and field athletes' historical competition performance data, and the effectiveness of the evaluation for individual track and field athletes' performance is yet to be verified. The experimental data are all track and field athletes' performance, and the generality of the prediction for other non-track and field sports is also yet to be verified. The next step will be to further explore the effectiveness of the model in evaluating the performance of athletes in a wider range of sports, to verify the generality of the model in evaluating athletes' performance, and to expand the scope of the application.

## Figures and Tables

**Figure 1:** Performance evaluation results of the 10 groups of 200m sprinters.

**Figure 2:** Estimation accuracy of the performance of the 10 track and field sports.

**Figure 3:** Evaluation accuracy of the three methods.

**Figure 4:** Evaluation efficiency of the three methods.

**Figure 5:** Comparison of the error evaluation indexes of the three methods.

**Table 1:** Variable declaration.

*I *_1_	Competition ranking
*I *_2_	Race time
*I *_3_	Age
*I *_4_	Gender
*I *_5_	The training time
*I *_6_	BMI
*I *_7_	Blood pressure

**Table 2:** KMO and Bartlett's test.

KMO sampling suitability quantity	0.592	
Bartlett sphericity test	The approximate chi-square	952.82
	Degrees of freedom	26
	Significant	0

**Table 3:** Total variance explained.

Composition	Total	Percentage of variance of initial eigenvalue	Cumulate %	Total	Load square and percent variance	Cumulate %	Total	Rotational load square and percent variance	Cumulate %
1	1.98	28.28	28.28	1.98	28.28	28.28	1.70	24.41	24.41
2	1.53	21.90	50.19	1.53	21.90	50.19	1.35	19.35	43.77
3	1.00	14.29	64.49	1.00	14.29	64.49	1.30	18.70	62.48
4	0.88	12.58	77.08	0.88	12.58	77.08	1.02	14.60	77.08
5	0.65	9.33	86.41						
6	0.54	7.77	94.19						
7	0.40	5.80	100.00						

**Table 4:** Rotated factor matrix and score matrix.

Variable	Indicators	Rotation factor matrix				Factor scoring matrix			
		1	2	3	4	1	2	3	4
*I *_1_	Competition ranking	0.846	−0.018	0.008	−0.001	0.519	−0.028	−0.116	0.044
*I *_2_	Race time	0.868	0.077	0.113	0.011	0.516	0.029	−0.048	0.035
*I *_3_	Age	−0.155	0.855	−0.035	0.123	−0.096	0.674	−0.149	−0.031
*I *_4_	Gender	0.278	0.748	0.231	0.001	0.124	0.561	0.032	−0.129
*I *_5_	The training time	−0.146	0.207	0.798	0.173	−0.205	0.010	0.650	0.090
*I *_6_	BMI	0.334	−0.044	0.773	−0.108	0.083	−0.1465	0.612	−0.127

**Table 5:** Hosmer-Lemeshaw test.

Chi-square	Degrees of freedom	Significant
9.806	8	0.278

**Table 6:** Prediction accuracy.

	Assessment of conformity		Accuracy rate	
	0	1		
Actual qualification	0	412	64	86.6
	1	118	132	52.8
Overall percentage	74.9			

**Table 7:** Logistic regression analysis.

	B	Standard error	Wald	Degree of freedom	Significance	Exp (B)	95% confidence interval of EXP (B)	
							Lower limit	Upper limit
Gender	0.65	0.09	51.66	1	0	1.92	1.61	2.3
BMI	0.86	0.1	75.36	1	0	2.38	1.96	2.9
Age	0.67	0.09	49.18	1	0	1.97	1.63	2.38
Training time	0.38	0.09	17.32	1	0	1.47	1.22	1.76
Constants	-0.82	0.09	76.33	1	0	0.43		

## Data Availability

The labeled dataset used to support the findings of this study is available from the corresponding author upon request.
